# Prognostic variables for temporal lobe injury after intensity modulated‐radiotherapy of nasopharyngeal carcinoma

**DOI:** 10.1002/cam4.1291

**Published:** 2018-02-23

**Authors:** Mei Feng, Yecai Huang, Xigang Fan, Peng Xu, Jinyi Lang, Dian Wang

**Affiliations:** ^1^ Department of Radiation Oncology Sichuan Cancer Hospital and Institute Sichuan Cancer Center School of Medicine University of Electronic Science and Technology of China Chengdu China; ^2^ Rush University Medical Center of Chicago Medical University Chicago Ilinois

**Keywords:** Biological effective dose, fraction size, nasopharyngeal carcinoma, radiation dose tolerance, radiation‐induced temporal lobe injury

## Abstract

To determine predictive factors for temporal lobe injury (TLI) in nasopharyngeal carcinoma patient (NPC) treated with intensity‐modulated radiation therapy (IMRT). A total of 695 NPC cases treated with IMRT were retrospectively analyzed. TLI was diagnosed on MRI images. Volume‐dose histograms for 870 evaluable temporal lobes were analyzed, and the predictive factors for the occurrence of TLI was evaluated. Receiver operating characteristic curve (ROC) and Logistic regression analysis was used to determine volume‐dose parameters that predict temporal lobe injury (TLI). Univariate and multivariate analysis were used to analyze the predictive factors for TLI. The radiation dose‐tolerance model of temporal lobe was calculated by logistic dose‐response model. The median follow‐up time was 73 months. A total of 8.5% patients were diagnosed with TLI. Among all the volume‐dose parameters, logistic regression model showed D2cc (the dose Gray delivered to 2 cubic centimeter volume) was an only independent predictive factor. Multivariate analysis showed D2cc of temporal lobe, fraction size of prescription, T stage, and chemotherapy were the independent predictive factors for TLI. Logistic dose‐response model has indicated the TD_5/5_ and TD_50/5_ of D2cc are 60.3 Gy and 76.9 Gy, respectively. D2cc of temporal lobe, fraction size of prescription, T stage, and chemotherapy were the possible independent predictive factors for TLI after IMRT of NPC. Biologic effective doses (TD_5/5_ and TD_50/5_) of D2cc are considered to prevent TLI.

## Introduction

Nasopharyngeal carcinoma (NPC) is a type of disease with distinct epidemiology, anatomy, and histopathology characteristics. It often occurred in China and southeast Asia, with the incidence rates in a range of 15 and 50 per 100,000 in southern provinces of China 1. Radiotherapy (RT) with or without chemotherapy is a mainstay in the treatment of NPC 2. Given the proximity of temporal lobes to NPC, temporal lobe injury (TLI) is one of serious late complications that affects memory 3, neurocognitive functions 3, physical functions 4, emotion 4, language 3, and the quality of life in survivors 4. In an era of 2D radiotherapy, the reported rate of TLI ranges from 3‐40% 5, 6, 7. Recent advancement of dose‐delivering technologies such as intensity‐modulated radiation treatment (IMRT) allows normal adjacent structures including temporal lobes to be spared from high‐dose radiation, which indeed led to reduction in incidence of radiation‐induced temporal lobe injury that varied from 4.6 to 16% 8, 9, 10.

In 1991, Emami first described the dose constraint of the brain. The dose ≥60 Gy delivered to 1/3 of whole brain volume was found to be predictive for ≥5% incidence at 5 years (TD_5/5)_ 11. Quantitative Analysis of Normal Tissue Effects in the Clinic (QUANTEC) reported the relationship between the radiation dose and incidence of TLI. Based on 2D radiotherapy, for fractionated RT with a fraction size of <2.5 Gy, an incidence of radiation injury of 5 and 10% is predicted to occur at a biologically effective dose of 120 Gy (range, 100–140) and 150 Gy (range, 140–170), respectively. For twice‐daily fractionation, a steep increase in toxicity appears to occur when the biologically effective dose is >80 Gy. For daily large fraction sizes (≥2.5 Gy), the incidence and severity of toxicity is unpredictable 12. Lee previously reported that incidence rate of TLI was estimated to be 5% at 10 years when temporal lobe received 64 Gy (equivalent dose) based on 2D radiation therapy 6. Of important notice, is that these data were created from conventional radiotherapy, and some heterogeneous factors such as different target volumes, endpoints, sample sizes, and irradiated brain regions would affect the clinical outcome.

However, in the modern era of IMRT, the reports about the TLI induced by IMRT or chemotherapy‐IMRT were relatively limited. Su and coworkers reported that a total of 4.6% patients were diagnosed with TLI among 870 NPC at a median follow‐up of 40 months. Of interest, TLI was not observed in T1‐2 patients, the incidence rates were 3.1 and 13.4% in T3 and T4 patients, respectively. The Dmax and D1cc in injured temporal lobes (TLs) are greater than that in normal TLs. The 5‐year incidence of TLI in patients with Dmax 64–68 Gy or D1cc 52–58 Gy is reported to be <5% based on this relatively short follow‐up 13.

Apparently, previously recommended dose constraints for radiation‐induced brain injury from QUANTEC are not adequately applied to IMRT of NPC. The dose constraints for TLI are urgently needed for NPC patients treated with IMRT. In this report, we conducted a retrospective analysis of 695 NPC treated with IMRT to determine predictive factors for TLI.

## Materials and Methods

### Patient selection

A total of 695 NPC patients treated with definitive IMRT in our institution were retrospectively reviewed and analyzed to determine predictive factors for TLI from June 2004–June 2009. All patients had a pathology‐proven NPC and had a local disease or locoregional disease (stage I–IV*a* + *b*) according to the UICC 7th TNM staging system, prior to definitive IMRT. Recurrence patients were excluded from our study. The basic characteristics such as age, gender, hypertension, diabetes, blood lipid, chemotherapy, target therapy and et al. were recorded carefully in Table 1. The study was approved by the ethics committee of our institution.

**Table 1:** Basic characteristics for 695 patients

Items	No.
Gender	
Male	540
Female	155
Age	
≥50	246
<50	449
T stage (UICC 7th)	
T1	21
T2	203
T3	239
T4	232
N stage (UICC 7th)	
N0	78
N1	253
N2	275
N3	89
TNM (UICC 7th)	
I	4
II	135
III	267
IV*a* + *b*	289
Diabetes	
Yes	26
No	669
Hypertension	
Yes	32
No	663
Smoking	
Yes	279
No	416
Alcoholism	
Yes	288
No	387
Chemotherapy	
Yes	532
No	163
Target therapy	
Yes	147
No	548
Cholesterol	
≥5.18 mmol/L	172
<5.18 mmol/L	523
Triglycerides	
≥1.70 mmol/L	183
<1.70 mmol/L	512

### Treatment

#### Radiotherapy protocol and temporal lobe contour

Radiation planning was designed and optimized using the CORVUS 3.4–4.2 inverse treatment planning system. The IMRT plan was implemented through dynamic intensity‐modulated coplanar arc irradiation using a multileaf collimator (Nomos mimic). The neck and shoulder thermoplastic mask was used to fix the patients. The target volumes were outlined according to the International Commission on Radiation Units and Measurements (ICRU) 50 and 62. The prescribed doses were as follows: 66–76 Gy for gross tumor volumes of the nasopharynx (GTVnx) (2.0–2.25 Gy/f), 66–70 Gy for positive neck lymph nodes (GTVln‐R/L) (2.0–2.2 Gy/f), 60–66 Gy for high‐risk clinical target volume (CTV1) (1.9–2.0 Gy/f), 54–60 Gy for low‐risk clinical target volume (CTV2) (1.8–1.9 Gy/f) and 50–54 Gy for lymphatic drainage regions (CTVln) (1.7–1.8 Gy/f), in 30‐33 fractions. All the patients received radiation to the lymph node drainage areas in the lower neck using ^60^Co split‐field techniques or 6 MV X‐ray split‐beam techniques with a prescription dose of 46–50 Gy 14. X‐ray was used to evaluate the setup errors before treatment delivery. The patients were treated with one fraction daily over 5 days per week. The dose limits for each normal organ were followed according to the Radiation Therapy Oncology Group protocol 0225 (RTOG0225). The whole process of IMRT was carried out according to an institutional treatment protocol previously described 14.

The temporal lobe (TL) delineated in the original treatment plan were reviewed, and was found that original TL contours did not include the areas that overlapped the tumor target volumes such as CTV and PTV, due to an inherent limitation of the Corvus system. For purpose of this study, we re‐delineated the entire TL and obtained the following dosimetric parameters: Dmax, Dmean, D0.1cc (the dose Gray to 0.1cc of the TL volume), D0.5cc, D1cc, D2cc, D3cc, D5cc, D10cc, D15cc, and D20cc.

#### Chemotherapy

Of the 695 patients, 163 patients received radiotherapy alone, while 532 received concurrent chemoradiotherapy with cisplatin 80 mg/m^2^ every 3 weeks for 2–3 cycles. Among 532 patients, 86 patients received 2–3 cycles of neoadjuvant chemotherapy combined with concurrent chemoradiotherapy. 47 patients received concurrent chemoradiotherapy combined with 1 to 2 cycle of adjuvant chemotherapy. The neoadjuvant chemotherapy regimen was TPF, and the adjuvant chemotherapy regimen was cisplatin.

#### MRI protocol

MRI brain was performed using a 1.5‐Tesla system (Signa CV/i; General Electric Healthcare, Chalfont St. Giles, United Kingdom), To diagnose TLI, our neuroradiologists examine the area from the suprasellar cistern to the inferior margin of the sternal end of the clavicle using a head‐and‐neck combined coil. T1‐weighted fast spin‐echo images in the axial, coronal, and sagittal planes (repetition time, 500–600 msec; echo time, 10–20 msec), and T2‐weighted fast spin‐echo MRI in the axial plane (repetition time, 4000–6000 msec; echo time, 95–110 msec) were obtained before injection of contrast material. After intravenous injection of gadopentetate dimeglumine (0.1 mmol/kg body weight Gd‐DTPA, Magnevist; Bayer‐Schering, Berlin, Germany), spin‐echo T1‐weighted axial and sagittal sequences and spin‐echo T1‐weighted fat‐suppressed coronal sequences were performed sequentially, using similar parameters to before injection. The section thickness was 5 mm with a 1 mm inter‐slice gap for the axial plane, and 6 mm with a 1 mm inter‐slice gap for the coronal and sagittal planes.

All brain MRI images were centrally reviewed by two neuroradiologists, Each MR was first independently reviewed. For those with any disagreement, a joint review was then performed with a consensus report as the final report for this study analysis. Diagnostic criteria for TLI were as follows: (1) white matter lesions, defined as areas of finger‐like lesions of increased signal intensity on T2‐weighted images; (2) contrast‐enhanced lesions, defined as lesions with or without necrosis on post‐contrast T1‐weighted images with heterogeneous signal abnormalities on T2‐weighted images; (3) cysts, round or oval well‐defined lesions of very high signal intensity on T2‐weighted images with a thin or imperceptible wall as previously reported 15. Recurrence or metastasis involved in TL was excluded from this study analysis.

### Follow‐up

The duration of follow‐up was calculated from the completion of IMRT to either the day of death or the day of last examination. All the patients were follow‐up every 3 months in the first years, every 6 months in the second year and every 12 months in the following years. Nasopharyngeal mirror, endoscopic examination, detailed physical examination and MRI were performed during follow‐up. Follow‐up MRI of the nasopharynx and/or neck was performed every 6–12 months, or whenever tumor recurrence was suspected or neurologic signs or symptoms occurred. The latency of TLI was measured from the day of IMRT completion to the date of MRI diagnosis.

### Statistical analysis

SPSS 19.0 was used for statistical analysis. Actuarial survival rates were calculated using the Kaplan–Meier method. Student's *t* test was used for comparing the dose between TLI and non‐TLI group. Receiver operating characteristic curve (ROC) was used for screening volume‐dose parameters to predict TLI. Logistic multiple stepwise regression was used for predicting the TLI rate from the physical and biological equivalent dose of the 11 volume‐dose parameters. For prognostic factor of TLI, long‐rank test was used for univariate analyses, and Cox proportional hazard model was used for multivariate analyses. TLI. The response variable was defined by classifying each temporal lobe depending on whether changes on MRI images. Dose and volume response curves were calculated with the nonlinear regression model using the logistic dose‐response model as below 16:

(1) $$P\left(X_{1},\;\;X_{2}\ldots X_{m}\right)=\frac{e^{\left(b_{0}\;\;+\;\;b_{1}^{*}X_{1}\;\;+\;\;b_{2}^{*}X_{2}\;\;+\;\;\ldots +b_{m}^{*}X_{m}\right)}}{1+e^{-(b_{0}\;\;+\;\;b_{1}^{*}X_{1}\;\;+\;\;b_{2}^{*}X_{2}\;\;+\;\;\ldots \;\;+\;\;b_{m}^{*}X_{m})}}$$

In the equation, b stands for the regression coefficient, *X*_1_, *X*_2_…*X*_m_ stand for the value of different volume‐dose parameters. Both physical dose and biological equivalent dose (BED) of temporal lobe were established. BED was calculated by linear quadratic model (${\text{EQD}}_{2}=D_{1}^{*}\left(\frac{d_{1}+\alpha /\beta }{2+\alpha /\beta }\right),\;\alpha /\beta =3$). The criterion for statistical significance was set at *α* = 0.05, and *P* values were determined from two‐sided tests.

## Results

Of the 695 patients, there were 21, 203, 239, and 232 patients for T1, T2, T3, and T4, respectively, according to UICC 7th staging system. The basic characteristics were summarized in Table 1. The median follow‐up time was 73 months (22–108). Fifty‐nine patients (8.49%) were diagnosed with TLI based on MRI images (Fig. 1). The median time of patients diagnosed with TLI was 38 months after completion of radiation (22–55 months). The incidences of TLI are 8.49% (59/695) in all patients. There was no TLI observed in T1 or T2 stage patients. Seventeen patients had some clinical symptoms including headaches, memory deterioration, emotion disorder, and et al. The other 41 patients did not complaint about any particular discomforts and exhibited obvious signs.

**Figure 1:** Typical MRI images for RITLI during follow up. RITLI, radiation‐induced temporal lobe injury. (A) Both temporal lobes showed decreased signal intensity on T1‐weighted image, especially for right temporal lobe; (B) Both temporal lobes showed increased signal intensity on T2‐weighted image; (C) Both temporal lobes showed contrast‐enhanced irregular lesions on T1‐weighted image in the axial plane; (D) Both temporal lobes showed contrast‐enhanced irregular lesions on T1‐weighted image in the sagittal plane.

### Dosimetric analysis of temporal lobes

In our study, the longest latency of TLI is 55 months, so the 59 patients with TLI all occurred within 60 months after IMRT. Of the 59 patients with TLI, 22 were diagnosed with bilateral TLI, and these 44 injured temporal lobes were included in this study. The other 37 patients were unilateral TLI, and 26 of the 37 patients who developed unilateral TLI within 60 months after IMRT were followed up for at least 60 months, so these 37 injured temporal lobes were included, and the uninjured temporal lobes in these 26 patients were considered as normal lobes for dose analysis. The 377 of 636 patients without TLI were followed up for at least 60 months and underwent MR imaging examinations at least once during the first 60 months of follow‐up to exclude TLI. Therefore, the actual incidence of TLI at 5 years is analyzed in 436 patients. Eighty‐one injured temporal lobes and 780 normal temporal lobes were enrolled in dosimetric analysis.

All 81 injured lobes containing TLI lesions received the maximal dose of each dosimetry planning in a range of 74.56 to 84.32 Gy. The dose of temporal lobe (Dmax, D0.1cc, D0.5cc, D1cc, D2cc, D3cc, D5cc, D10cc, D15cc, D20cc, and Dmean) in TLI group were significantly higher than that of non‐TLI group (*P* < 0.05) (Table 2). For ROC curve, the AUC of D2cc (0.856 ± 0.025) was the greatest one among all the parameters (Table 3).

**Table 2:** The radiation dose of temporal lobe in the patients with TLI or non‐TLI

Volume‐dose parameters	TLI (mean ± SD Gy)	Non‐TLI(Gy) (mean ± SD Gy)	*P* value
Dmax	80.36 ± 6.74	73.82 ± 5.45	0.000
D0.1cc	78.91 ± 6.00	71.22 ± 6.02	0.000
D0.5cc	77.08 ± 6.11	68.52 ± 6.40	0.000
D1cc	75.24 ± 6.34	65.83 ± 7.02	0.000
D2cc	72.88 ± 6.90	62.20 ± 7.92	0.000
D3cc	70.73 ± 7.47	59.11 ± 8.60	0.000
D5cc	66.60 ± 8.78	53.79 ± 9.62	0.000
D10cc	57.19 ± 11.53	44.04 ± 10.40	0.000
D15cc	49.31 ± 12.84	37.01 ± 10.86	0.000
D20cc	42.82 ± 13.33	31.78 ± 10.85	0.000
Dmean	29.11 ± 8.54	25.34 ± 15.78	0.039

TLI, temporal lobe injury.

**Table 3:** ROC curve for TLI in NPC patients with different volume‐dose parameters of temporal lobe

Volume‐dose parameters	Area under curve	SE	95%CI
Dmax	0.798	0.03	0.739–0.857
D0.1cc	0.817	0.028	0.762–0.871
D0.5cc	0.835	0.027	0.783–0.887
D1cc	0.846	0.026	0.796–0.897
D2cc	0.856	0.025	0.806–0.906
D3cc	0.854	0.026	0.804–0.905
D5cc	0.843	0.027	0.789–0.896
D10cc	0.808	0.031	0.748–0.868
D15cc	0.776	0.032	0.713–0.838
D20cc	0.748	0.034	0.682–0.814
Dmean	0.65	0.033	0.585–0.716

CI, confidence interval.

### Univariate and multivariate analysis of TLI

For the univariate analysis, T stage, chemotherapy, diabetes, physical dose of temporal lobe (D2cc), biological dose of temporal lobe (D2cc) and fraction size of prescription was the substantial predictive factors. For the multivariate analysis, only T stage, chemotherapy, D2cc of temporal lobe, and fraction size of prescription were independent risk factors for TLI (Table 4).

**Table 4:** Univariate and multivariate analysis of 436 patients for TLI

Items	No. of non‐TLI (%)	No. of TLI (%)	Univariate analysis		Multivariate analysis	
			*x* ^2^	*P*	HR	*P*
Gender						
Male	308 (70.64%)	50 (11.47%)	0.322	0.570	–	–
Female	69 (15.83%)	9 (2.06%)				
Age						
≥50	160 (36.70%)	30 (6.88%)	1.467	0.226	–	–
<50	217 (49.77%)	29 (6.65%)				
T stage (UICC 7th)						
T1	19 (4.36%)	0 (0.0%)	37.167	0.000	2.525	0.000
T2	112 (25.69%)	0 (0.0%)				
T3	135 (30.96%)	22 (5.04%)				
T4	111 (25.46%)	37 (8.49%)				
Diabetes						
Yes	14 (3.21%)	5 (1.15%)	2.775	0.096	1.552	0.080
No	363 (82.26%)	54 (12.39%)				
Hypertension						
Yes	20 (4.59%)	4 (0.92%)	0.213	0.644	–	–
No	357 (81.88%)	55 (12.61%)				
Smoking						
Yes	157 (36.01%)	24 (5.50%)	0.020	0.899	–	–
No	220 (50.46%)	35 (8.03%)				
Alcoholism						
Yes	161 (36.93%)	28 (6.42%)	0.469	0.493	–	–
No	216 (49.54%)	31 (7.11%)				
Chemotherapy						
Yes	301 (69.04%)	55 (12.61%)	6.096	0.014	–	–
No	76 (17.43%)	4 (0.92%)				
Target therapy						
Yes	80 (18.35%)	17 (3.90%)	1.070	0.192	–	–
No	297 (68.12%)	42 (9.63%)				
Cholesterol						
≥5.18 mmol/L	92 (21.10%)	20 (4.59%)	2.409	0.121	–	–
<5.18 mmol/L	285 (65.37%)	39 (8.94%)				
Triglycerides						
≥1.70 mmol/L	102 (23.40%)	15 (3.44%)	0.069	0.792	–	–
<1.70 mmol/L	275 (63.07%)	44 (10.09%)				
D2cc (BED) (temporal lobe side)						
≥60.3 Gy	340 (38.99%)	69 (7.91%)	52.545	0.000	3.755	0.000
<60.3 Gy	451 (51.72%)	12 (1.38%)				
D2cc (radiation dose fraction)						
≥2 Gy	366 (41.97%)	69 (7.91%)	44.508	0.000	2.819	0.009
<2 Gy	425 (48.74%)	12 (1.38%)				

TLI, temporal lobe injury; HR, hazard ratio.

### Dose‐response analysis

For the physical dose of the volume‐dose parameters, Logistic multiple stepwise regression analysis showed only D2cc was the independent prognostic factor for TLI among these 11 volume‐dose parameters (Dmax, D0.1cc, D0.5cc, D1cc, D2cc, D3cc, D5cc, D10cc, D15cc, D20cc, and Dmean) (*P* = 0.000, Odds ratio = 1.299) (Table 5), so the original equation was simplified as equation: $P\left(X_{\mathrm{PD}}\right)=\frac{e^{\left(b_{0}+X^{*}b_{1}\right)}}{1+e^{-(b_{0}+X^{*}b_{1})}}$,in which *X*_PD_ stands for physical dose of D2cc and *P*(*X*_PD_) stands for predicted incidence rate of TLI when the D2cc is *X*_PD_. *b*0 and *b*1 of D2cc were −19.147 (95%CI: −23.387, −14.907) and 0.261 (95%CI: 0.200, 0.322). Therefore, TD5/5 was 61.97 Gy (95%CI: 60.735, 63.193) and TD50/5 was 73.26 Gy (95%CI: 71.98, 74.46) (Fig. 2A).

**Table 5:** Logistic multiple stepwise regression analysis results of volume‐dose parameters for TLI

Factor	B	SE	*Wald*	*Sig*	Exp(B)	95%CI for Exp(B)	
						Lower	Upper
D2cc	0.261	0.031	71.516	0.000	1.299	1.222	1.308
Constant	−19.147	2.163	78.341	0.000	0.000	–	–
D2cc (BED)	0.177	0.021	72.394	0.000	1.193	1.146	1.243
Constant	−13.602	1.498	82.416	0.000	0.000	–	–

TLI, temporal lobe injury; CI, confidence interval.

**Figure 2:** Dose‐response analysis of D2cc in temporal lobe for RITLI. (A) physical dose of D2cc in temporal lobe for RITLI; (B) biological equivalent dose of D2cc in temporal lobe for RITLI. RITLI, radiation‐induced temporal lobe injury.

For the biologically equivalent tolerance dose (BED) of the volume‐dose parameters, logistic multiple stepwise regression analysis also showed D2cc was the only independent parameter that could predict TLI (*P* < 0.001, OR = 1.193, 95%CI: 1.146, 1.243). The original equation was simplified as equation: $P\left(X_{\mathrm{BED}}\right)=\frac{e^{\left(b_{0}+X^{*}b_{1}\right)}}{1+e^{-(b_{0}+X^{*}b_{1})}}$, in which *X*_BED_ stands for BED of D2cc and *P*(*X*_BED_) stands for predicted incidence rate of TLI. *b*0 and *b*1 of D2cc were −13.602 (95%CI: −16.538, −10.666) and 0.177 (95%CI: 0.136, 0.208). Therefore, TD5/5 was 60.3 Gy (95%CI: 59.7, 61.5) and TD50/5 was 76.9 Gy (95%CI: 75.7, 78.2) (Fig. 2B).

## Discussion

Temporal lobe injury (TLI) is one of the most serious late effects after the definitive radiotherapy of NPC. Results from this study and other few studies 9, 13, 17 have demonstrated that incidence rates of TLI in patients treated with modern IMRT are indeed significantly reduced, in comparison with previous reports in the era of conventional radiotherapy 11, 12. Similar to the previous report 13, we observed TLI in patients treated with T3–T4 NPC, but not in patients with T1‐2 NPC. However, the incidence of TLI was 8.49% in patients with T3‐4 in our study at a median follow‐up of 73 months, which was higher than 6.7% observed in a previous study at a median follow‐up of 40 months 13. This difference could be related to a relatively short follow‐up time in the previous study 13 (median follow‐up of 40 months vs. 73 months in this study), and in this study, we noticed a median time to diagnose TLI was 38 months. The above difference might explain a high incidence rate of TLI in patients with NPC in this study.

The precise mechanism that causes TLI remains unknown, but TLI is likely to be associated with the volume and dose of TL irradiated. Su found that IMRT with rV40 <10% or aV40 <5cc, and a Dmax < 68 Gy or D1cc < 58 Gy for the TL was less likely to develop TLI 13. Among several volume‐dose and volume‐dose parameters, Sun reported only D0.5cc was predictive for TLI (D0.5cc < 69 Gy) 18. In this study, we noticed the area under cures (AUC) of D2cc was the predictable factor for TLI among all the dosimetric parameters. Based on the dose‐response analysis (Figure 3), we noticed the close correlation between incidence rate of TLI and D2cc of temporal lobe, which indicates the importance of AUC of D2cc to predict TLI. The D2cc < 60.31 Gy for TD5/5 and 76.85 Gy for TD50/5 thresholds should be considered as the constraint dose of TL in the IMRT of NPC. However, we are still not able to define specific TLI areas that are associated with radiation dose, even though we carefully review the CT dosimetry and MRI.

Radiation‐induced injury of temporal lobe is a highly complex and multifactorial process. Radiation tolerance may vary depending on patient‐ and tumor‐specific characteristics, as well as treatment modifications. Our multivariate analysis showed T stage, chemotherapy, D2cc of temporal lobe and fraction size of prescription were the independent risk factors for TLI. Similarly, Zeng reported the T category, chemotherapy and Dmax of temporal lobe were the significant factors affecting the risk of temporal lobe injury 18. Furthermore, Lee 11 reported the 10‐year actuarial incidence of TLN was 4.6% for patients irradiated to 60.0 Gy with 2.5 Gy per fraction, and up to 18.6% for those irradiated to 50.4 Gy with 4.2 Gy per fraction. In a prospective trial, 25 patients are treated by IMRT for a total of 70 Gy with 2.34 Gy per fraction to GTV, and TLI becomes one of the common late complications with a high incidence at 12% 19. Our results showed that fraction size of prescription (>2 Gy) was the independent risk factors for TLI, which was consistent with the previous studies. Besides the volume‐dose parameters of radiation, the age, chemotherapy, diabetes, and hypertension were reportedly predictive factors for TLI 20, 21. Results of our study confirmed that chemotherapy was indeed the prognostic factor for TLI, but others (diabetes, hypertension, alcohol and smoke, blood lipid, and target therapy) were not found to be independent risk factors for TLI in this study. In this study, 76.5% patients received chemotherapy.

Shortcoming of this study is retrospective nature. The follow‐up time might not be enough for NPC, even though, to the best of our knowledge, this study has the longest median follow‐up time (73 months) among the literature reports on IMRT of NPC. In addition, current MRI diagnosis of TLI is not completely defined, even though we have assigned two neuroradiologists to independently review each MRI. The NTCP model established in this study warrants further validation in a separate external validation cohort, and the D2cc e constraints based on this NTCP model should be treated with caution before use.

In a conclusion, results from this study have suggested that radiation dose of temporal lobe, T stage, fraction size of prescription, and chemotherapy were the independent predictive factors for TLI. D2cc was an important parameter for TLI. TD5/5 and TD50/5 of D2cc are 60.3 Gy and 76.9 Gy, these biological effective dose thresholds should be considered in IMRT planning of NPC.

## Conflicts of Interest

There is no conflict of interest.
